# Distinctive Gut Microbiota Alteration Is Associated with Poststroke Functional Recovery: Results from a Prospective Cohort Study

**DOI:** 10.1155/2021/1469339

**Published:** 2021-12-07

**Authors:** Yini Dang, Xintong Zhang, Yu Zheng, Binbin Yu, Dijia Pan, Xiaomin Jiang, Chengjie Yan, Qiuyu Yu, Xiao Lu

**Affiliations:** ^1^Division of Neurological Rehabilitation, Department of Gastroenterology, The First Affiliated Hospital of Nanjing Medical University, Jiangsu, China; ^2^Department of Gastroenterology, The First Affiliated Hospital of Nanjing Medical University, Jiangsu, China; ^3^Department of Rehabilitation Medicine, The First Affiliated Hospital of Nanjing Medical University, Jiangsu, China

## Abstract

**Objectives:**

Functional prognosis is potentially correlated with gut microbiota alterations following the dysregulation of the gut-microbiota-brain axis after stroke. This study was designed to explore the poststroke alterations of gut microbiota and potential correlations between gut microbiota and global functions.

**Methods:**

A total of thirty-eight patients with stroke and thirty-five healthy demographics-matched controls were recruited. Their fecal DNAs were extracted, and the V3-V4 regions of the conserved bacterial 16S RNA were amplified and sequenced on the Illumina MiSeq platform. Microbial composition, diversity indices, and species cooccurrence were compared between groups. Random forest and receiver operating characteristic analysis were used to identify potential diagnostic biomarkers. Relationships between discriminant bacteria and poststroke functional outcomes were estimated.

**Results:**

Higher alpha diversity of gut microbiota was observed in poststroke patients as compared to the healthy controls (*p* < 0.05). Beta diversity showed that microbiota composition in the poststroke group was significantly different from that in the control group. Relative abundance of nine genera increased significantly in poststroke patients, while 82 genera significantly decreased (*p* < 0.05). The accuracy, specificity, and susceptibility of the optimal model consisted of the top 10 discriminant species were 93%, 100%, and 86%, respectively. Subgroup analysis showed that bacterial taxa abundant between subacute and chronic stroke patients were overall different (*p* < 0.05). The modified Rankin scale (mRS) (*r* = −0.370, *p* < 0.05), Fugl-Meyer assessment (FMA) score (*r* = 0.364, *p* < 0.05), water swallow test (WST) (*r* = 0.340, *p* < 0.05), and Barthel index (BI) (*r* = 0.349, *p* < 0.05) were significantly associated with alterations of distinctive gut microbiota.

**Conclusions:**

The gut microbiota in patients with stroke was significantly changed in terms of richness and composition. Significant associations were detected between alterations of distinctive gut microbiota and global functional prognosis. It would facilitate novel treatment target selection in the context of stroke while the causal relationships between distinctive gut microbiota alterations and functional variations need to be further verified with well-designed studies.

## 1. Introduction

Stroke has been reported to be the major global health issue with an annual incidence of 258 per 100,000 person-years worldwide [1]. Patients suffering from stroke impose a heavy medical and economic burden on both society and the family [2]. With the medical advances in interventions for stroke (e.g., intravenous thrombolysis and endovascular treatment), the survival rate has been significantly improved while the disability rate increases [3]. Although medical treatment for stroke is essential for competing with the life-threatening condition in the acute phase, sequels left by stroke (e.g., motor dysfunction, cognitive dysfunction, or swallowing dysfunction) may subsequently impact the patients' health-related quality of life and increase the burden on families and society [4, 5]. This indicates that attention should be, to some extent, moved forward to foresee the long-term functional prognosis; therefore, early modification of corresponding interventions can be provided. According to the literature review, several factors which may impact the poststroke functional recovery have been reported including age, gender, and admission National Institutes of Health Stroke Scale (NIHSS) score [6–8]. Nonetheless, these consolidated factors revealed only the individualized properties which could ever be changed or influenced [9–11]. Upon this condition, exploring novel functional prognosis-associated factors, which may potentially serve as treatment targets, becomes the most warranted task in front of clinicians.

Among the several newly proposed theories, investigation into the role of the “gut-microbiota-brain axis” in regulating neurological function has rapidly increased over the past decades [12, 13]. Dysregulation of the gut-microbiota-brain axis has been increasingly linked to the pathophysiology of stroke [14, 15]. Interactions across gut microbiota and poststroke functional outcomes were mainly observed in animal models [16, 17]. Nonetheless, the role of human gut microbiota is indeed somewhat different from animals [18]. The following concerns were the limited knowledge regarding the role human gut microbiota played with neural plasticity and the following prognostic changes. A few cross-sectional studies have explored the composition of gut microbiota in patients with stroke compared with healthy demographics-matched controls. For instance, dysbiosis of short-chain fatty acid- (SCFA-) producing bacteria and SCFAs in patients with acute ischemic stroke was previously observed [19]. Alterations in trimethylamine-producing gut bacteria were proved to be associated with stroke [20]. However, these studies provided single-time point observations (e.g., data collected only at the acute phase) or enrolled only subtypes of stroke (e.g., middle cerebral artery occlusion). In addition, clinical trials remain limited in their ability to show the potential links between the gut microbiome, systematic and neural responses, and global functional changes in the context of stroke.

Based on the above concerns and rationales, we conducted this study to answer the following two clinical questions: (1) should there be any discrepancies of gut microbiota in terms of either richness or composition between poststroke patients and healthy controls and (2) should there be certain potential correlations between gut microbiota alteration and global functions including general disability, physical function, swallowing function, and activity of daily living (ADL)? With the elaboration of the above two questions, our understanding regarding the role the “gut-microbiota-brain axis” played in the development of stroke would be improved followed by promoting novel treatment target selection in the context of stroke.

## 2. Materials and Methods

### 2.1. Study Design and Patient Enrollment

The current cohort study was conducted at the First Affiliated Hospital of Nanjing Medical University from 04 July 2020 to 29 January 2021. It was approved by the Committee of Institutional Ethics (Institutional Review Board, 2018-SR-339), and all participants provided written informed consent prior to participation.

The inclusion criteria were as follows: (1) ischemic or hemorrhagic stroke confirmed with computed tomography (CT) or magnetic resonance imaging (MRI), (2) aged 18 yr or older, (3) able to verbally respond to the instructions, and (4) with stable vital signs (systolic blood pressure of 120-180 mmHg, heart rate of 50-100/min, body temperature < 37.5°C, and blood oxygen saturation > 92%) [21, 22]. Patients were excluded if (1) diagnosed with the transient ischemic attack (TIA), (2) with severe cognitive and mental dysfunctions (Montreal Cognitive Assessment < 26) [4, 23], and (3) currently enrolled in another trial or participated in a clinical trial within 6 months [24, 25]. Matched healthy controls were also enrolled according to age, nutritional status (body mass index (BMI)), and geographical area.

### 2.2. Functional Assessment and Sample Collection

Demographic information including age, gender, BMI, blood pressure, smoking history, alcohol intake, physical activities, stroke subtype, medical history, and family history were collected according to a face-to-face interview or from electronic medical records. Functional assessments were performed by a research assistant with validated and reliable scales. Specifically, stroke severity was assessed with NIHSS score; a higher score indicates greater stroke severity [26]. Modified Rankin scale (mRS) was used to measure the degree of disability and dependence in daily activities. mRS score ranges from 0 (no symptom) to 6 (death) with an unfavorable outcome scored 3-6 and a favorable outcome scored 0-2 [27, 28]. ADL was evaluated with Barthel index (BI) ranging 0-100, with a lower score indicating higher dependence [29]. Upper or lower extremity motor function was assessed with Fugl-Meyer assessment (FMA) score such that a lower score indicates worse motor function [30, 31]. Swallowing function was assessed with the water swallow test (WST); a higher grade indicates a higher risk of aspiration [32, 33]. Fecal samples were collected from both groups and immediately immersed in a solution and stored at -80°C for subsequent DNA extraction.

### 2.3. DNA Extraction and Illumina Sequencing

DNAs extracted from the fecal samples were used to amplify the V3-V4 region of the 16S rRNA gene targeted with primer set 341 F/806R. This action was performed to determine the gut bacterial community structure. The amplified products were further subjected to the library preparation and sequenced on the Illumina MiSeq platform according to the manufacturer instructions (Illumina technologies, USA).

### 2.4. Bioinformatics and Statistical Analysis

The raw fastq files obtained from the Illumina sequencing machine were quality filtered with trimmomatic, vsearch, etc. High-quality sequence was used for community structure analysis through the QIIME pipeline. Operational taxonomic unit (OTU) picking was carried out with UCLUST closed reference method, and the representative OTUs were assigned taxonomy using UCLUST classifier by using the SILVA database (Version 132) as a reference dataset.

Alpha and beta diversity indicates the gut microbial diversity of the different patients in the poststroke or control group assessed within (alpha diversity) and across (beta diversity) samples. Alpha diversity estimation was computed using the ace and Shannon indexes. Beta diversity was estimated with principal coordinates analysis (PCA), Bray-Curtis, and partial least squares discrimination analysis (PLS-DA). The Wilcoxon test was used to identify significantly differential OTUs (*p* < 0.05) for further analysis. Significant differences in the relative abundance of associated taxa between groups were further determined with linear discriminant analysis integrated with effect size (LEfSe). Random forest models (R3.4.1, randomForest 4.6-12 package) were performed to develop a predictive model. Receiver operating characteristic curve (ROC) and area under the curve (AUC) were used to evaluate the accuracy of models (R3.3.0, pROC package).

Continuous variables were presented as means and standard deviations. Categorical variables were demonstrated as numbers and percentages. Continuous nonnormal distribution variables were compared between groups with the Wilcoxon rank sum test. Fisher's exact test was used to compare intergroup differences for categorical variables. Correlations between discriminant bacterial and functional assessments were estimated with the Spearman correlation analysis. Differences between groups were considered significant as *p* values less than 0.05.

## 3. Results

### 3.1. Demographic and Clinical Characteristics

A number of 38 subjects with clinical diagnosis of poststroke patients (aged 59.18 ± 15.34; male/female 25/13) were recruited, including 18 subacute and 20 chronic patients. We followed the guideline and defined the subacute stroke as duration of stroke for less than 30 days while chronic stroke as duration of stroke for more than 30 days [34]. Meanwhile, 35 age- and sex-matched healthy individuals (aged 59.36 ± 15.30; male/female 23/12) were also enrolled. Detailed demographic and clinical characteristics of stroke patients and controls are shown in Tables 1 and 2.

### 3.2. Alterations of Gut Microbiota Composition in Poststroke

Venn diagram displayed 210 common OTUs between groups (Figure 1(a)). However, 133 unique OTUs were detected in the poststroke group and 36 in the control group, respectively (Figure 1(a)). Alpha diversity analysis showed that poststroke patients were characterized with higher richness and diversity than the controls (ace indexes 43335.18 ± 7270.54*vs.*29467.57 ± 6848.03; Shannon indexes 13.50 ± 0.78*vs.*11.03 ± 0.79, *p* < 0.05, Figures 1(b) and 1(c)). Results of Bray-Curtis and PCA were also demonstrated in Figures 1(d) and 1(e). In addition, PLS-DA showed that microbiota composition in the poststroke group significantly differed from that in the control group (Figure 1(f)).

At the family level, *Enterococcaceae*, *Lachnospiraceae*, *Enterobacteriaceae*, and *Helicobacteraceae* were significantly enriched while *Neisseriaceae*, *Porphyromonadaceae*, *Flavobacteriaceae*, *Weeksellaceae*, *Cardiobacteriaceae*, and *Pasteurellaceae* were markedly depleted in the poststroke group (Figure 2(a)). At the genus level, the abundance of 9 genera, including *Lachnoclostridium*, *Flavonifractor*, *Lactobacillus*, *Enterococcus*, and *Enterobacter*, was significantly elevated in the poststroke group. However, the abundance of 82 genera, including *Blautia*, *Faecalibacterium*, *Roseburia*, *Fusicatenibacter*, and *Prevotella*, was found to be significantly decreased in the poststroke group (Figure 2(b) and Table 3). Among these significantly differentiated genera, 18 genera (e.g., *Blautia*, *Fusicatenibacter*, *Ruminococcus*, *Romboutsia*, *Prevotella*, and *Roseburia*) were SCFA-producing bacteria (Figure 2(c)). According to the bacteria from the Human Oral Microbiome (HOM, Version 13) database, oral colonizers (including 26 genus and 67 species) presented significantly differentiated abundance in the poststroke group (Figure 2(d)). As compared to the controls, an abundance of 25 species elevated while 146 decreased in the poststroke group (Table 4).

### 3.3. Gut Microbiota-Based Prediction of Poststroke Functional Recovery

The linear discriminant analysis (LDA) and distribution diagram analysis (LDA score > 3.5) showed alteration of the microbiota with higher genus *Fusobacterium*, *Lactobacillus*, *Enterococcus*, *Veillonella*, *Megamonas*, and *Escherichia* levels in the poststroke group (Figures 3(a) and 3(b)). However, genus *Blautia*, *Prevotella*, *Fusicatenibacter*, *Roseburia*, *Faecalibacterium*, *Ruminococcus*, and *Neisseria* levels were significantly enriched in the control group (Figures 3(a) and 3(b)).

To explore potential biomarkers for the prediction of poststroke functional variation, a random forest model was constructed based on the differentiated species (relative abundance > 0). Tenfold cross-validation analysis showed the AUCs of 95% (Figure 3(c)). As per the above analysis, the accuracy, specificity, and susceptibility of the optimal model consisted of the top 10 species (Figure 3(d)) were 93%, 100%, and 86%, respectively.

### 3.4. Disease Duration-Dependent Variation of Gut Microbiota

Genera cooccurrence networks between groups based on the Pearson correlation analysis are demonstrated in Figures 4(a) and 4(b). Positive correlations were demonstrated between *Aggregatibacter* and *Neisseria*, *Porphyromonas*, *Corynebacterium* and between *Capnocytophaga* and *Leptotrichia*, *Porphyromonas*, *Neisseria* (rho ranged 0.87-0.97, *p* < 0.05) in the control group, while between *Pseudobutyrivibrio* and *Roseburia*, *Flavonifractor* and *Lachnoclostridium*, and *Fusicatenibacter* and *Pseudobutyrivibrio* (rho ranged 0.66-0.76, *p* < 0.05) in the poststroke group. The subacute patients showed positive correlations between *Fusicatenibacter* and *Pseudobutyrivibrio*, *Flavonifractor* and *Lachnoclostridium*, *Fusicatenibacter* and *Roseburia*, and *Pseudobutyrivibrio* and *Roseburia* (rho ranged 0.67-0.80, *p* < 0.05) (Figure 4(c)). In the chronic subgroup, we observed that *Pseudobutyrivibrio* and *Roseburia*, *Aggregatibacter* and *Neisseria*, *Aggregatibacter* and *Porphyromonas*, *Capnocytophaga* and *Leptotrichia*, *Capnocytophaga* and *Pseudobutyrivibrio* (rho ranged 0.53-0.81, *p* < 0.05) were positively correlated (Figure 4(d)).

In addition, the bubble plots and LEfSe (LDA score > 2.5) showed significantly increased/decreased bacterial taxa abundant in both subacute and chronic stroke patients (Figures 4(e) and 4(f)). Genus (e.g., *Megasphaera*, *Paraprevotella*, and *Howardella*) and species (e.g., *Bacteroides thetaiotaomicron*, *Lactobacillus mucosae*, and *Parabacteroides johnsonii*) were significantly enriched in subacute patients, while *Lactococcus*, *Barnesiella*, *Bifidobacterium kashiwanohense*, *Bacteroides salyersiae*, and *Lactococcus garvieae* were significantly enriched in the chronic subgroup. According to the alpha diversity analysis, no significant differences were detected between the subacute and chronic groups (Figures 4(g) and 4(h)).

### 3.5. Correlation between Differentiated Bacterial Genus with Poststroke Functional Variation

Several bacterial taxa (e.g., *Barnesiella*, *Blautia*, *Coprococcus*, *Enterococcus*, and *Lactococcus*) demonstrated significantly differentiated abundance in the poststroke group. Significant positive correlations were observed between variations of *Prevotella* and FMA-UE (*r* = 0.328, *p* < 0.05), *Enterococcus* and FMA-LE (*r* = 0.364, *p* < 0.05), *Lactococcus* and WST (*r* = 0.340, *p* < 0.05), and *Prevotella* and BI (*r* = 0.349, *p* < 0.05), respectively (Figure 5). Significant negative correlations, between variations of *Butyricicoccus* and FMA-LE (*r* = −0.333, *p* < 0.05) and *Enterococcus* and mRS (*r* = −0.370, *p* < 0.05), were also detected (Figure 5).

## 4. Discussion

In the current study, we firstly observed the higher alpha diversity and beta diversity of gut microbiota in poststroke patients as compared to those in the healthy controls, indicating the poststroke community richness and composition of gut microbiota differed from healthy controls. Afterward, a panel of microbiota was identified as biomarkers (e.g., *Aggregatibacter segnis* and *Neisseria mucosa*) to distinguish disease status. Furthermore, sensitivity analysis was performed to explore the gut microbiota alteration according to the length of stroke from onset (e.g., subacute and chronic) [34]. Significantly variated gut microbiota composition was observed along with the progress of stroke. Finally, we also demonstrated that general disability level, motor function either for upper limb or lower limb, swallowing function, and ADL were significantly associated with alterations of distinctive gut microbiota. Taken together, our results further provided evidence to support the point of view that gut microbiota varies following stroke. The hypothesized linkage between gut microbiota alterations and functional prognosis was preliminary observed while the causal relationships underlying these observations need to be further verified with well-designed animal and clinical studies.

Upon the great complexity of gut microbiota and huge heterogeneity of individual properties, studies into the role of gut microbiota on stroke were started with animal experiments to avoid the interference of confounding factors on outcome observation. By using two distinct mouse models of stroke, the overgrowth of microbiota (e.g., *Firmicutes*, *Bacteroidetes*, and *Actinobacteria*) was previously identified as biomarkers of poststroke microbiota dysbiosis, indicating that microbiota dysbiosis could serve as instruments to guide diagnosis and prognosis prediction of stroke [35, 36]. Due to the discrepancy of gut microbiota between humans and animals, several studies on humans were initiated to better understand the poststroke gut microbiota alterations. For instance, a novel parameter termed as Stroke Dysbiosis Index (SDI) was proposed to discriminate stroke patients from healthy controls with AUCs ranging 74.9%-84.3% [37]. This is the first compound biomarker proposed to account for the poststroke gut microbiota alterations. However, the accuracy of the discriminative ability was not as high as in the current study. Here, we used the random forest model with which a panel of 10 significantly variated gut microbiota was detected with AUCs ranging 93%-95%. The accuracy of the discriminative ability was further improved with our model, and it provided reliable results for the following analysis.

The poststroke gut microbiota alterations can be explained by several proposed theories. For instance, central stress responses induced reduction of gastrointestinal motility that may lead to bacterial overgrowth [38]. The autonomic nervous system has also been implicated in mediating the effects of stroke on dysbiosis [39]. Specifically, poststroke stress responses may lead to imbalanced activities of the autonomic nervous system which in turn increase intestinal permeability via releasing corticotropin and glucocorticoid hormones and consequently lead to gut bacterial translocation [40, 41]. In addition, mouse model transplanted with poststroke fecal microbiota showed higher expression of the inflammatory T cells Th1 and Th17 indicating that systemic metabolic, immunologic, and inflammatory responses may play roles in the poststroke gut microbiota alterations [35, 42]. To elaborate on the underlying mechanisms of the above responses, our results preliminarily demonstrated a decreased abundance of SCFA-producing bacteria (e.g., *Blautia*, *Fusicatenibacter*, and *Ruminococcus*) in patients with stroke. Liu and colleagues also found that a deficiency of SCFA-producing bacteria was significantly associated with poststroke cognitive impairment [43]. Transplantation of fecal microbiota rich in SCFAs was found to be effective in the improvement of stroke [44]. This protective effect was related to the enhancement of gut barrier integrity and attenuating systemic inflammation, which may improve function of the blood-brain barrier, decrease cerebral edema, and attenuate brain injury [45]. This further verified the role of SCFAs in the development and prognosis of stroke; it may serve as a novel treatment target for stroke. With the clarification of specific mechanisms in animal steps, this flow also indicated that it needs to be moved forward to clinical circumstances for better facilitating the application of achievements from human trials.

In addition, poststroke variation of specific bacteria may have subsequent influences on regional organ responses. According to our results, an increased abundance of opportunistic pathogens was observed in patients with stroke. The potential role of opportunistic pathogens, such as *Enterobacteriaceae*, was reported to be associated with intestinal epithelial dysfunction [46]. Overgrowth of the *Enterobacteriaceae* may lead to inflammation exacerbation or exogenous pathogen invasion while internal homeostasis was disrupted [47]. These biological communications between the human body and gut microbiota may highlight the novel targets of stroke management. We also observed decreased potential probiotics. Based on the literature review, probiotics or a combination of probiotics and prebiotics could alter the composition of the gut microbiome followed by neuroinflammatory changes and cytokine releases. On the other hand, probiotics was demonstrated to increase brain-derived neurotrophic factor (BDNF) and inhibit apoptosis [48]. Taken together, the specific bacteria may influence the prognosis of stroke. Identification of this distinctive gut microbiota may contribute to the development of innovative treatment targets.

Although we observed the above promising variations of gut microbiota followed by the explanation of the potential internal mechanisms of subsequent consequences, the next question is that “should there be certain potential correlations between gut microbiota alterations and global functions” based on the newly discovered variations of gut microbiota across healthy and stroke status. The abundance of *Christensenellaceae* and *Ruminococcaceae* has been reported to be positively correlated with NIHSS score and mRS while *Enterobacter* was negatively correlated [49]. Our results preliminarily demonstrated that global functions, including general disability level, motor function, swallowing function, and ADL, were significantly associated with alterations of distinctive gut microbiota. There has been published a number of studies on exploring the relationship between microbiome and prognosis after stroke. Li et al. reported a negative correlation of *Enterobacter* with mRS score at one month [49]. Similar results have been also observed in our study. Apart from that, *Prevotella* was found to be correlated with motor function and ADL. The potential explanation would be that *Prevotella* was considered to be associated with mucosal inflammation, which may impact poststroke functional recovery due to the immune response [50, 51]. However, the next challenge in front of us is to answer the question “whether the alterations of distinctive gut microbiota are the causes or consequences of poststroke neural plasticity.” This would further improve our understanding of the role the “gut-microbiota-brain axis” played in the development of stroke and facilitate the treatment target selection.

The current study has several strengths and limitations. Firstly, we applied the random forest model to estimate the distinctive gut microbiota across stroke patients and healthy controls. This action further improved the accuracy of discriminative ability in detecting distinctive gut microbiota as compared to the previous studies. Nonetheless, the results should be further verified and validated in larger samples so that several subgroup analyses in terms of microbiota discrepancy could be performed. In addition, the current study preliminarily reported the potential correlations between gut microbiota alterations and global functions while the underlying mechanisms and the causal relationships between the gut microbiota, systematic and neural responses, and global functional changes need to be further investigated to build up the whole picture of the role the “gut-microbiota-brain axis” played in the context of stroke.

## 5. Conclusion

To sum up, poststroke gut microbiota was significantly modified as compared to healthy controls. The main characteristics of the stroke-induced shift in composition were the decreased abundance of SCFA-producing bacteria and the increased abundance of opportunistic pathogens. Significant associations were detected between alterations of distinctive gut microbiota and poststroke functional prognosis. A better understanding of the precise interactions between gut microbiota, systematic and neural responses, and global functional changes may be helpful in the identification of novel therapeutic targets to improve poststroke functional recovery.

## Figures and Tables

**Figure 1:** Diversity of gut microbiota. (a) Venn diagram of common OTUs. (b, c) Alpha diversity is estimated with the ace and Shannon index. (d–f) Beta diversity was estimated with Bray-Curtis, PCA, and PLS-DA. OTU: operational taxonomic unit; PCA: principal coordinates analysis; PLS-DA: partial least squares discrimination analysis. ^∗^*p* < 0.05.

**Figure 2:** Alteration of gut microbiota composition. (a) Composition of gut microbiota at a family level. (b) Heatmap of gut microbiota composition at the genus level. (c) Venn diagram of the significantly different bacterial genus in poststroke and SCFA-producing bacterial genus. (d) Venn diagram of significantly different bacterial genus/species in poststroke and oral bacterial genus/species. SCFAs: short-chain fatty acids.

**Figure 3:** Identification of microbiota-based biomarkers for stroke. (a) Cladograms generated from LEfSe. (b) LDA scores for the differentially abundant bacterial taxa (LDA score > 3.5). Red bars indicate taxa enriched in the poststroke group; green bars indicate taxa enriched in the control group. (c) ROC analysis for random forest model. (d) List of 10 discriminant bacterial taxa based on random forest model. LDA: linear discriminant analysis; ROC: receiver operating characteristic curve; AUC: area under the curve.

**Figure 4:** Subgroup analysis of gut microbiota in stroke. (a) Correlation network in the control group. (b) Correlation network in the poststroke group. (c) Correlation network in the subacute patients. (d) Correlation network in chronic patients. (e) OTU bubble plot indicated differences in genus level between subgroup of poststroke patients and control group. (f) LDA scores for differentiated bacterial taxa are abundant between the subacute and chronic patients (LDA score > 2.5). Red bars indicate taxa enriched in the chronic group; green bars indicate taxa in the subacute group. (g, h) Alpha diversity is estimated with the ace and Shannon index. OTU: operational taxonomic unit; LDA: linear discriminant analysis. ^∗^*p* < 0.05.

**Figure 5:** Correlations between differentiated bacterial genus and variations of functional status. BI: Barthel index; FMA-LE: Fugl-Meyer assessment lower extremity scale; FMA-UE: Fugl-Meyer assessment upper extremity scale; WST: water swallow test; mRS: modified Rankin scale; NIHSS: National Institutes of Health Stroke Scale. ^∗^*p* < 0.05.

**Table 1:** Summary of demographic and clinical characteristics.

	Poststroke (*n* = 38)	Control (*n* = 35)	*p* value
Age in year, mean (SD)	59.18 (15.34)	59.36 (15.30)	0.902
Gender, *n* (%)			0.995
Male	25 (65.79)	23 (65.71)	
Female	13 (34.21)	12 (34.29)	
Height in centimeter, mean (SD)	168.53 (6.95)	167.03 (6.83)	0.375
Weight in kilogram, mean (SD)	69.21 (11.33)	66.66 (8.02)	0.274
BMI in kg/m^2^, mean (SD)	24.25 (2.87)	23.95 (3.07)	0.594
SBP in mmHg, mean (SD)	127.61 (15.21)	126.00 (10.72)	0.607
DBP in mmHg, mean (SD)	79.13 (10.07)	79.94 (8.16)	0.708
Glucose in mmol/L, mean (SD)	4.52 (0.55)	4.39 (0.62)	0.373
Total cholesterol in mmol/L, mean (SD)	3.38 (1.08)	3.39 (0.70)	0.964
Triglycerides in mmol/L, mean (SD)	1.44 (0.52)	1.45 (0.50)	0.944
Occupation, *n* (%)			0.403
Full time or part time	19 (50.00)	15 (42.86)	
Layoffs	0 (0)	1 (2.86)	
Retired	17 (44.74)	13 (37.14)	
Self-employed	1 (2.63)	4 (11.43)	
Others	1 (2.63)	2 (5.71)	
Marriage status, *n* (%)			0.343
Unmarried	0 (0)	1 (2.86)	
Married	36 (94.74)	30 (85.71)	
Widowed	2 (5.26)	2 (5.71)	
Divorced	0 (0)	1 (2.86)	
Others	0 (0)	1 (2.86)	
Education, *n* (%)			0.201
Primary school or less	0 (0)	1 (2.86)	
Secondary school	11 (28.95)	4 (11.43)	
High school	20 (52.63)	24 (68.57)	
College/university	7 (18.42)	5 (14.28)	
Postgraduate	0 (0)	1 (2.86)	
Smoking status, *n* (%)			0.131
Nonsmoker	23 (60.53)	20 (57.14)	
Current smoker	13 (34.21)	8 (22.86)	
Previous smoker	2 (5.26)	7 (20.00)	
Alcohol intake, *n* (%)			0.438
No drinking	16 (42.11)	20 (57.14)	
Light drinking	13 (34.21)	9 (25.72)	
Heavy drinking	9 (23.68)	6 (17.14)	
Regular physical activities, *n* (%)			0.187
Yes	6 (15.79)	10 (42.86)	
No	32 (84.21)	25 (57.14)	

SD: standard deviation; BMI: body mass index; SBP: systolic blood pressure; DBP: diastolic blood pressure.

**Table 2:** Summary of clinical characteristics in patients with subacute or chronic stroke.

	Subacute (*n* = 18)	Chronic (*n* = 20)	*p* value
Type of stroke, *n* (%)			0.018
Hemorrhage stroke	4 (22.22)	13 (65.00)	
Ischemic stroke	13 (72.22)	7 (35.00)	
Hemorrhagic transformation	1 (5.56)	0 (0)	
Duration of stroke (day), median (IQR)	27 (15)	93 (111)	<0.001
Medical history, *n* (%)			0.821
Ischemic stroke	1 (5.56)	0 (0)	
Hemorrhage stroke	1 (5.56)	1 (5.00)	
Subarachnoid hemorrhage	0 (0)	0 (0)	
Stroke not classified	0 (0)	0 (0)	
Hypertension	5 (27.78)	9 (45.00)	
Diabetes mellitus	3 (16.67)	2 (10.00)	
Dyslipidemia	0 (0)	0 (0)	
Atrial fibrillation	1 (5.56)	1 (5.00)	
Coronary heart disease	1 (5.56)	1 (5.00)	
Congenital heart disease	0 (0)	0 (0)	
Valvular heart disease	0 (0)	0 (0)	
Other types of heart disease	0 (0)	0 (0)	
Peripheral arterial disease	0 (0)	0 (0)	
Others	0 (0)	1 (5.00)	
Hypertension history in year, mean (SD)	11.50 (5.82)	8.33 (4.47)	0.254
Diabetes mellitus history in year, mean (SD)	7.67 (2.52)	7.50 (3.54)	0.954
Family history, *n* (%)			—
Stroke	0 (0)	0 (0)	
Coronary heart disease	0 (0)	0 (0)	
Hypertension	1 (5.56)	1 (5.00)	
Diabetes mellitus	0 (0)	0 (0)	
Dyslipidemia	0 (0)	0 (0)	
NIHSS score, mean (SD)	9.44 (4.66)	8.55 (5.89)	0.602
mRS, *n* (%)			0.846
0-2	5 (27.78)	5 (25.00)	
3-6	13 (72.22)	15 (75.00)	
BI, mean (SD)	34.44 (19.77)	45.00 (27.338)	0.149
FMA-UE score, mean (SD)	19.56 (21.38)	24.05 (17.44)	0.584
FMA-LE score, mean (SD)	16.33 (10.09)	18.84 (10.30)	0.626
WST, *n* (%)			0.895
Grade 1	13 (72.22)	13 (65.00)	
Grade 2	2 (11.11)	3 (25.00)	
Grade 3	1 (5.56)	1 (5.00)	
Grade 4	2 (11.11)	2 (10.00)	
Grade 5	0 (0)	1 (5.00)	

SD: standard deviation; IQR: interquartile range; NIHSS: National Institutes of Health Stroke Scale; mRS: modified Rankin scale; BI: Barthel index; FMA-UE: Fugl-Meyer assessment upper extremity scale; FMA-LE: Fugl-Meyer assessment lower extremity scale; WST: water swallow test.

**Table 3:** Top 20 significantly increased/decreased genus in the poststroke group.

Increased genus			Decreased genus		
OTU	Average difference	Adjusted *p* values	OTU	Average difference	Adjusted *p* values
Enterococcus	3.12	0.001	Blautia	-1.35	<0.001
Lactobacillus	2.92	0.003	Erysipelatoclostridium	-2.45	<0.001
Enterobacter	2.51	0.007	Pseudobutyrivibrio	-2.47	<0.001
Helicobacter	1.36	0.001	Neisseria	-6.92	<0.001
Kluyvera	1.21	0.025	Haemophilus	-2.39	<0.001
Flavonifractor	0.99	0.004	Chryseobacterium	-1.63	<0.001
Anaeroplasma	0.76	0.024	Actinobaculum	-1.75	<0.001
Lachnoclostridium	0.76	0.018	Filifactor	-1.99	<0.001
Pectobacterium	0.60	0.039	Selenomonas	-2.04	<0.001
			Treponema	-2.05	<0.001
			Catenibacterium	-2.06	<0.001
			Lachnoanaerobaculum	-2.25	<0.001
			Caproiciproducens	-2.26	<0.001
			Lautropia	-2.28	<0.001
			Mannheimia	-2.41	<0.001
			Campylobacter	-2.60	<0.001
			Anaerostipes	-1.45	0.002
			Fusobacterium	-2.40	0.003
			Lachnospira	-2.40	0.041
			Coprococcus	-0.82	0.041

OTU: operational taxonomic unit.

**Table 4:** Top 20 increased/decreased species with the significant difference in the poststroke group.

Increased species			Decreased species		
OTU	Average difference	Adjusted *p* values	OTU	Average difference	Adjusted *p* values
Enterococcus raffinosus	1.60	0.008	Erysipelatoclostridium ramosum	-2.45	<0.001
Enterobacter ludwigii	1.71	0.012	Blautia obeum	-2.64	<0.001
Veillonella tobetsuensis	1.64	0.013	Anaerostipes butyraticus	-2.64	<0.001
Enterococcus viikkiensis	1.39	0.014	Fusicatenibacter saccharivorans	-3.01	<0.001
Lactobacillus apodemi	0.96	0.015	Gemmiger formicilis	-3.37	<0.001
Staphylococcus gallinarum	0.95	0.015	Leptotrichia goodfellowii	-2.20	<0.001
Lachnoclostridium urinimassiliense	0.68	0.015	Neisseria dentiae	-1.61	<0.001
Shigella boydii	1.18	0.015	Neisseria cinerea	-1.67	<0.001
Lactobacillus fermentum	1.88	0.017	Mannheimia granulomatis	-1.72	<0.001
Escherichia vulneris	1.28	0.019	Actinobaculum massiliense	-1.75	<0.001
Staphylococcus xylosus	1.04	0.024	Neisseria wadsworthii	-1.77	<0.001
Anaeroplasma abactoclasticum	0.75	0.024	Capnocytophaga granulosa	-1.93	<0.001
Helicobacter ganmani	0.72	0.024	Campylobacter showae	-1.93	<0.001
Megasphaera micronuciformis	1.95	0.026	Porphyromonas gingivalis	-1.96	<0.001
Enterobacter kobei	0.88	0.030	Lachnoanaerobaculum orale	-1.98	<0.001
Lactobacillus casei	1.04	0.034	Filifactor alocis	-1.99	<0.001
Lactococcus garvieae	1.05	0.039	Catenibacterium mitsuokai	-2.06	<0.001
Lactococcus formosensis	0.89	0.039	Cardiobacterium valvarum	-2.14	<0.001
Lactobacillus murinus	0.88	0.039	Campylobacter gracilis	-2.18	<0.001
Kluyvera ascorbata	0.87	0.039	Faecalibacterium prausnitzii	-1.69	0.039

OTU: operational taxonomic unit.

## Data Availability

The data used to support the findings of this study are available from the corresponding author upon request.
